The article "Artificial Intelligence in Cardiology and Atherosclerosis in the Context of Precision Medicine: A Scoping Review" was published in 2024. Journal: Appl Bionics Biomech.

# Artificial Intelligence in Cardiology and Atherosclerosis in the Context of Precision Medicine: A Scoping Review

**DOI:** 10.1155/2024/2991243

**Published:** 2024-04-30

**Authors:** Oliwia Kolaszyńska, Jacek Lorkowski

**Affiliations:** ^1^Department of Internal Medicine, Asklepios Clinic Uckermark, Am Klinikum 1, 16303, Schwedt/Oder, Germany; ^2^Department of Orthopedics, Traumatology and Sports Medicine, Central Clinical Hospital of the Ministry of Internal Affairs and Administration, 137 Woloska Street, Warsaw 02-507, Poland; ^3^Faculty of Engineering and Physical Sciences, University of Surrey, Guildford, UK

## Abstract

Cardiovascular diseases remain the main cause of death worldwide which makes it essential to better understand, diagnose, and treat atherosclerosis. Artificial intelligence (AI) and novel technological solutions offer us new possibilities and enable the practice of individually tailored medicine. The study was performed using the PRISMA protocol. As of January 10, 2023, the analysis has been based on a review of 457 identified articles in PubMed and MEDLINE databases. The search covered reviews, original articles, meta-analyses, comments, and editorials published in the years 2009–2023. In total, 123 articles met inclusion criteria. The results were divided into the subsections presented in the review (genome-wide association studies, radiomics, and other studies). This paper presents actual knowledge concerning atherosclerosis, in silico, and big data analyses in cardiology that affect the way medicine is practiced in order to create an individual approach and adjust the therapy of atherosclerosis.

## 1. Introduction

The perception of a human being as a structure with numerous mathematical dependencies has been developed over the centuries. First examples can be found in antiquity and among Pythagoreans who investigated the nature of numbers and their relationship with the world exhaustively. It is suspected that the world-famous first computer, the Antikythera mechanism, was designed by Pythagoreans [1] and that the Lycurgus Cup made by the ancient Romans is the first example of the use of nanotechnology [2]. Today, the most important synthesis seems to have been published in “The fractal geometry of nature” by Kirkby [3]. It introduces the concept of fractals, connects dependencies that can be described by the Fibonacci Sequence, and have been discovered over a long time, such as the Julia set, the Cantor set, the Hausdorff dimension, the Sierpiński triangle, and the Sierpiński carpet. Similarly, the chromatin cell architecture is considered to be fractal, as well as other biological structures and processes [4]. Their description demands artificial intelligence (AI) because of its complexity which corresponds more to quantum than classical physics. Quantum physics, quantum computing, and AI are currently dynamically evolving fields of science. AI is a perfect candidate for quantum computing as its assumptions are mostly based on probabilistic elements, require huge amounts of data, and significantly increase the efficiency of already existing systems [5]. This is why quantum machine learning (ML) is gaining popularity.

Cardiovascular disease (CVD) remains the leading cause of death [6]. Together with the Fourth Industrial Revolution and AI solutions, new approaches are being proposed to expand the actual risk stratification, diagnosis, and treatment of CVD; to provide therapy tailored to an individual in the context of precision medicine; and to explain possible interactions affecting the pathophysiology of atherosclerosis. The amount of data collected to screen and then diagnose and treat an individual requires AI. In the case of atherosclerosis, optimal treatment is based not only on the experience of the physician but also on the individual characteristics of the atherosclerotic lesions in the body.

This paper presents current knowledge on atherosclerosis, in silico, and big data analysis with AI, and AI performing other human functions that can be used in everyday medical practice to achieve better outcomes, speed up workflow, reduce costs, improve diagnostics and treatment solutions, and better understand a complex atherosclerotic disease. As atherosclerosis remains the leading cause of death, optimal diagnosis and treatment of patients are of paramount importance. Analyzed data will be used in the context of precision medicine and its potential application in personalized therapy.

## 2. Methodology

The study was performed based on the Preferred Reporting Items for Systematic Reviews and Meta-Analyses (PRISMA) protocol.

### 2.1. Inclusion Criteria

The main inclusion criteria were the presence of AI solutions and the connection of the topic with personalized medicine.

### 2.2. Exclusion Criteria

Studies performed on animals and concerning cardiovascular risk stratification as well as those with no possibility of verifying applied methods were excluded from this review.

### 2.3. Search Methodology

PubMed and MEDLINE databases were searched using the Boolean operators “AND” and “OR.” The following commands were used “artificial intelligence” OR “AI” AND “atherosclerosis” (*n* = 4,458); “artificial intelligence” OR “AI” AND “atherosclerosis” AND “cardiology” AND “GWAS” (*n* = 110); “artificial intelligence” OR “AI” AND “cardiology” AND “precision medicine” (*n* = 352); “artificial intelligence” OR “AI” AND “cardiology” AND “radiomics” (*n* = 31). For “artificial intelligence” OR “AI” AND “atherosclerosis,” an additional filter was used to include papers published in the last 10 years. Two researchers conducted searches independently of each other. No automation tools were applied: (1) articles with similar contents were chosen by the publication date—the newest were included; (2) articles written by the same author and concerning the same issue—the newest were included. The results were divided into subsections presented in the review. The inclusion and exclusion criteria as well as organization of articles are presented in Table 1.

The authors identified 4,951 records. One hundred fifty nine records were removed due to duplication and 4,335 due to inconsistency with the topic. As of 10 January 2023, 457 articles were included for further analysis. Of the 457 articles, 11 were performed on animals, 73 involved cardiovascular risk stratification, 225 were inconsistent with the topic, and 18 were reviews. There were seven articles in which the authors could not verify the methods and decide whether they met the inclusion criteria. These articles were excluded. Finally, 123 studies were included. All articles have been divided into the following subsections presented in the article: genome-wide-association study, radiomics, and other applications.

The process is presented in Figure 1.  Figure 2 presents an overview of the application of AI in the medical context.

## 3. Genome-Wide Associated Studies (GWAS) and Artificial Intelligence in Atherosclerosis

Genetics is a field of medicine that connects mathematics, physics, and biology. It is complicated character and the fact that the majority of traits are created by an interplay of various genes resulting in a particular phenotype makes it difficult to find a pattern for their distribution in a general population. A theory of infinitesimal model assumes that the continual discovery of new genes affecting particular trait contribute to a smaller causality in each of them [7]. Precision medicine's goal is to tailor an individualized therapy based on, among other things, genetic profiling, and to assess if there exists an increased risk for a particular disease or a severe variant. Tools used by precision medicine are genome-wide associated studies (GWAS) that enable the identification of single-nucleotide polymorphisms (SNPs), and exome sequencing. Surprisingly, these important particles of the human genome mostly reside in its noncoding part and are often not linked to particular genes. Therefore, it is difficult to determine the significance of some mutations [8, 9]. It was proven that many loci susceptible to particular disease fall within enhancers specific to disease-relevant types of cells, for example, the 1p13 locus, rs12740374, altering SORT1 gene hepatic expression with minimal effect in other cells [10]. However, it is still possible that even the most important loci have small effect sizes which explains only a part of genetic variation. This phenomenon is called the mystery of “missing heritability” and was partially solved by analyses concerning SNPs [11].

Not without meaning is the importance of AI as it enables the integration of all collected high-dimensional data based on multiomic studies. The number of analyses concerning CVDs, mostly caused by complex and heterogeneous factors like multiple genetic, environmental, and behavioral factors, is constantly growing. Not least because CVD is globally the leading cause of mortality and morbidity [6]. The nascent amount of data gathered by various institutions to improve the quality of healthcare, increase cost-effectiveness, workflow, and adopt rising precision medicine assumptions needs special measures, such as ML. In the light of these findings, new methods of big data analysis, such as variant-Set Test for Association using Annotation infoRmation (STAAR) or JACUSA software (implemented for detection of SNPs), have been proposed [12, 13].

It should be mentioned that most genetic studies are based on Mendelian randomization and GWAS. These are methods that do not fit into the strict definition of AI that exists today. They are used as hybrid methods, mostly in big data analysis, i.e., statistics or protein–protein interaction [14]. Yet, they yield such an amount of data that is hard and time-consuming to analyze without AI application. Nowadays, questions arise as to whether these newly described loci are of biological importance, and which mechanisms are connected with their action and disease-relevant function. Below we present the most relevant studies performing their analyses in silico or using AI approaches and big data analyses.

Studies of human atheroma plaques have been performed for years but have hardly resulted in the most important knowledge during recent years. Depuydt et al. [15] exhaustively analyzed the cellular landscape of human atheroma identifying 14 main cell populations with an in silico method. They found a predominance of T-cells in the lymphocyte population and confirmed that the CD4 + CD28 null line plays an important role in patients with CVD, as well as found pro- and anti-inflammatory cells, distinct endothelial cells (this can be proof for the endothelial to mesenchymal cell transition), and evaluated the cellular interplay within the plaque. The authors additionally integrated GWAS data to find cell-specific loci responsible for CVD and to determine potential individual targets for drug intervention. Single-cell RNA sequencing and cytometry by time of flight gave a new insight into the macrophage population within the plaque and their function [16]. Another study examined 7,000 human atherosclerotic cells and exploited GWAS as a source to reveal how specific cell types participate in particular diseases, identify cell- and tissue-specific enhancers, and genes that are likely to be influenced by the noncoding genome, describe transcription factors that could play an important role in smooth muscle cell differentiation, as well as describe superenhancers (defined as those driving the expression of genes important for cell identity and function) in lesion cell types, in the context of atherosclerosis [17].

Recent years have brought important knowledge of non-coding RNAs (ncRNAs) as cardiovascular risk factors and regulators of human cells. They can be divided into long non-coding RNAs (lncRNAs), micro-RNAs (miRNA), and small interference RNAs (siRNAs) [18, 19]. Imprinting represents epigenetic marks common to genes requisite for early development and growth of the placenta. Its loss leads to the expression of miRNA-regulated genes. MicroRNAs, small noncoding single-stranded molecules repressing gene expression at the posttranscriptional level, are not less important in the pathophysiology of atherosclerosis. An epigenomic study of altered DNA methylation was performed finding a hypomethylated imprinted chromosomal locus 14q32 encoding over 60 mRNAs and 70 snoRNAs. The most relevant seems to be the RTL-1 gene (RTL1AS encodes for the hsa-mir-431, -433, -127, -432, and -136) and has-mir-127 as both are upregulated in atherosclerotic plaques and may become potential drug targets [20]. Other studies try to identify new pharmacological targets for CVDs [21, 22]. The influence of monocyte ncRNA on the underlying cardiovascular disorders, including atherosclerosis, was evaluated in a study by Pérez-Sánchez et al. [23] gathering patients with antiphospholipid syndrome. Studies using AI to describe the pathophysiology of atherosclerosis have been performed, i.e., to analyze the impact of ncRNA on the immune response, and find out that the immune system and smooth muscle cell cytoskeleton dysregulation accelerate atherosclerosis progression [24].

Since 2007 and the breakthrough discovery of 9p21 locus by four independent groups of researchers, over 163 loci have been identified and another 300 are suspected to be connected with coronary artery disease (CAD) risk. They implicate the same pathways in atherosclerosis etiology-vascular tone, blood pressure, low-density lipoprotein (LDL-C), triglyceride-rich lipoproteins, inflammation, cellular migration, smooth muscle cell proliferation, and vascular remodeling, lipoprotein (a), neovascularization and angiogenesis, and NO/cGMP signaling. Moreover, a lot of CAD risk loci exhibit an association with other diseases and traits and are designated as pleiotropic. It is estimated that combined they are responsible for 30%–40% of CAD heritability but particular mechanisms remain unknown [25, 26].

Locus 8q24, containing the gene TRIB1, has been associated with the therapeutically beneficial lipid profile and seems to play a key role in plasma lipid homeostasis [27–29]. PHACTR1 gene regulation was proven to have a huge impact on the severity of vascular calcifications in a murine model [30] and the impact of genetic variation can be seen in vascular smooth muscle cells function [31].

A study by Meng et al. [32] presented potential key genes (C3AR1, CCR1, CCR2, CD33, CD53, CXCL10, CXCL8, CXCR4, CYBB, FCER1G, FPR2, ITGAL, ITGAM, ITGAX, ITGB2, and LILRB2) for atherosclerosis pathology that may become potential drug targets. Additionally, a thorough analysis indicated immunity, chemokines, and cell adhesion molecules as the most important biological factors in atherosclerosis.

In 2021, Levin et al. [33] presented a large study identifying 116 SNPs associated with stroke, 107 with CAD, and 105 with peripheral artery disease (PAD). In their study, authors suggest that smoking had an atherogenic effect in all the vascular beds as well as show that the genetic liability for smoking can influence other, already identified cardiovascular risk factors [33].

Lipoprotein A level is linked to atherosclerosis, although its atheroprotective role is still being discussed [34]. A study by Zekavat et al. [35] showed that knowledge of particular lipoprotein A genotype enables more specific CVD risk prediction and that the heritability is high in European and African American populations (75% and 85%, respectively). Recently, APOH was identified as a novel locus for lipoprotein A encoding ß2-glycoprotein I [36]. Another study performed GWAS analysis of 441,016 UK Biobank participants to find out that apolipoprotein B has the highest correlation with coronary heart disease of all studied lipid particles [37]. Holliday et al. [38] found an extensive genetic overlap between large artery atherosclerosis and small vessel ischemic stroke which suggests a potential shared genetic pathogenesis, based on GWAS of 12 389 ischemic stroke patients. Awan et al. [39] investigated genetics of familial hypercholesterolemia.

Among 8,536 patients of African and European ancestry with type 2 diabetes mellitus a GWAS study has been performed. Diabetic patients tend to have higher coronary artery calcification (CAC) and common carotid intima-media thickness (cIMT). The authors have identified a new locus rs8000449 near CSNK1A1L at 13q13.3 for association with CAC, two other loci have been confirmed for CAC and one for cIMT. Locis rs2891168 near CDKN2B-AS1 at 9p21 and rs11170820 near FLJ12825 at 12q13.13 for CAC; rs7412 near APOE at 19q13.32 for cIMT have been correlated with a CAD [40].

Last but not least is the analysis of big data described by Shendre et al. [41] who performed GWAS of 682 HIV-positive and 288 HIV-negative black women and measured carotid intima-media thickness to define whether European ancestry and SNPs may affect the cIMT. The study showed a possible influence of the local European ancestry on atherosclerosis, yet did not define particular SNPs associations with cIMT. Two SNPs within the ryanodine receptor (RYR3) gene were associated with cIMT among HIV patients treated with highly active antiretroviral therapy [42].  Table 2 presents studies included in this analysis.

## 4. Radiomics and Artificial Intelligence in Atherosclerosis

A standard in cardiologic procedures includes visualization of the heart, coronary arteries, and aorta with echocardiography, computed tomography, and magnetic resonance.

Echocardiography is a method of visual estimation of the heart—muscle, valves, and aorta—and it does not only depend on precise calculation. It owes its status as a basic diagnostic tool in cardiology mostly to modern AI-based solutions. The road from the PipieLined Image Processing Engine (PIPE) in 1985 through automated strain measurements 20 years later to the current multichamber automatic analyses has been long. ML was introduced to assess the ejection fraction (EF) and longitudinal strain [43, 44]. In heart failure (HF), ML was applied to diagnose HF with preserved EF, classify symptomatic, and asymptomatic patients using strain technology, predict hospitalization risk, exercise tolerance, E/e' measurements, define isolated diastolic dysfunction, and left ventricle filling pressure [45, 46]. Madani et al. [47] presented an algorithm to classify echocardiogram images with a 97.8% accuracy and no overfitting. No less important is the application of ML-based methods in the detection of wall motion abnormalities, assessment of the response of the cardiac muscle to the resynchronization therapy, prediction of major adverse cardiac events (MACEs) or coronary artery calcium (CAC), recognition, and assessment of valvular heart disease, classification of echocardiograms, differentiation of hypertrophic cardiomyopathy (HCM) and physiological hypertrophy of the athletes, or restrictive cardiomyopathy (RCM), and constrictive pericarditis [43, 48–51].

Yet, some limitations cannot be omitted. First, echocardiography is a subjective test. Second, the problem of repeatability is created by the fact that input data are highly dependent on the person performing an examination. Third, AI can detect and characterize valvular and anatomic pathology as well as enhance the quality of existing echocardiograms but is certainly unable to accurately assess all cardiac pathologies that could be noticed and described by a clinician [52].

The importance of cardiovascular computed tomography (CCT) has grown since the 1990s when it was used to assess stenotic regions of arteries and occlusion of bypass grafts. Nowadays, with new diagnostic methods and AI, it has become possible to create visual simulations helpful in planning surgeries, assessing postsurgical complications, predicting outflow tract obstruction, and other hemodynamic complications, or identifying the high-risk phenotype of left ventricular hypertrophy [53, 54]. Computational fluid dynamics (CFD) and finite element (FE) simulations have been used in transcatheter aortic valve replacement, transcatheter mitral valve implantation, thoracic endovascular aortic repair, left atrial appendage occlusion, and to assess myocardial strains [55–59]. All simulations have been helpful to make personal predictions and assumptions concerning treatment. However, ML does not need CFD or FE simulations to result in excellent outcomes.

Studies by Hu et al. [60] and Gupta et al. [61] proposed a radiomic tool to improve the diagnostic performance of cardiovascular computed tomography angiography (CCTA). Atkov et al. [62] diagnosed CAD based on clinical and laboratory data combined with SNPs and CCTA with 64%–94% accuracy. CT and AI solutions have been applied in the identification of hemodynamically significant coronary artery stenosis, also by computing fractional flow reserve (FFR) [63] which is arising as a noninvasive alternative in diagnosing chest pain. Recently, culprit lesions have been studied using ML models based on CCTA of 60 patients with an acute myocardial infarction. The authors have shown that culprit lesions and severe stenosis present some characteristic features [64].

ML–FFR was found to be a better tool than CCTA to detect and quantify CAC [44]. Interestingly, a performance test between CFD-FFR and ML-FFR was found to be equal [65]. Prediction of obstructive CAD was performed by Al'Aref et al. [66] based on 35,281 patients from the CONFIRM registry. ML was also applied in CCTA to assess volumes of ventricles and atria, detect plaques and identify culprit lesions in acute coronary syndromes (ACS), measure CAC, prepare and segmentation CT images, phenotype coronary plaques, and predict cardiovascular risk [43, 67–69]. As an alternative, a ML method with intravascular ultrasound (IVUS) was proposed to assess FFR in intermediate coronary lesions [70] or to classify the components of an atherosclerotic plaque [71]. Interestingly, the action connective matrixes have been developed to extract potentially invisible features from IVUS images and reduce the image noise [72].

In the recent years, the role of perivascular adipose tissue (PVAT) has been connected with an increased cardiovascular risk. Hypotheses concerning the influence of the inflammatory process within PVAT on worsened CVD outcomes have been broadly discussed in the literature [73]. Thus, it is of high importance to create appropriate and repetitive tools to assess the plaque-associated risk. Oikonomou et al. [74] presented an AI-based tool, the fat radiomic profile (FRP), to assess cardiovascular risk based on CT scans of periadventitial fat. The FRP enabled observation of changes that are dynamic and reversible, including fibrosis, vascularity, and tissue homogeneity. These factors influence adipose tissue health in obesity as well and altogether have created a noninvasive tool to assess the cardiovascular risk better than already established risk factors like age, sex, diabetes, systolic blood pressure, body mass index, obstructive CAD, total cholesterol level, high-density lipoprotein level, and Agatston calcium calcification score (CCS) [74]. A study by Commandeur et al. [75] proposed an AI approach to quantify epicardial and thoracic adipose tissue based on non-contrast CT scans. Eisenberg et al. [76] stated that the epicardial adipose tissue volume is positively correlated with an increased risk of major adverse cardiovascular events (MACE), while attenuation was inversely associated.

Cardiac magnetic resonance (CMR) was highly affected by technological advancements which have boosted its diagnostic and risk stratification capabilities [43]. According to the ESC guidelines, it is the gold standard to assess volumes, mass, and EF of both the left and right ventricles [77]. Together with ML, it was used to assess ventricular volumes, strain, filling, and ejection rate, predict an all-cause death in HF patients, analyze and describe cardiac structures, scars in HCM patients, diagnose HCM, differentiate HCM and hypertensive heart disease, diagnose pulmonary artery hypertension, predict outcomes in newly diagnosed pulmonary hypertension, segmentate, and diagnose carotid atherosclerosis [43, 77–82].

Another approach used CMR in patients with ST-elevation myocardial infarction (STEMI) and stated that radiomics could provide higher diagnostic accuracy for detecting microvascular obstruction [83] as well as become a new tool to predict MACEs [84]. However, the first clinical application of ML-based algorithms in everyday practice might be an algorithm estimating volumes of the left ventricle in CMR [62].

Although databases containing medical information are still being discussed in the ethical context of sensitive data, their need has been highlighted in many fields [85]. Also, nuclear cardiology expressed the proposition of building large image databases which could help to speed up the workflow, reduce costs, and create appropriate prognostic models [85, 86]. Artificial neural networks have been used to detect myocardial ischemia using 99mTc-methoxyisobutylolisonitryle myocardial perfusion images [86]. In the case of nuclear cardiology, AI has been applied to assess cardiac perfusion, predict obstructive CAD, early revascularization, and MACEs, as well as automatically localize the mitral valve plane to prevent image artifacts. Moreover, implemented methods can outperform current clinical approach results [62, 86–92].

The basic goal of radiomics is to present clinically important features incorporated in medical images. Implemented to support genomic data with an AI-based analysis yields precise radiogenomic results. Although it has mostly been applied with outstanding success in oncology, it can be implemented into practice in most medical disciplines, including cardiology [85, 92].  Table 3 presents studies included in this analysis.

## 5. Artificial Intelligence and Atherosclerosis in Other Studies

Zhao et al. [99] proposed a tool for ECG autodiagnosis of ST-elevation myocardial infarction (STEMI). His algorithm achieved results highly comparable with those achieved by an experienced cardiologist and better than medical doctors [99]. Similarly, a deep learning-based algorithm to recognize myocardial infarction by Makimoto et al. [100] was tested in comparison to physicians. Another idea from the Mayo Clinic enabled the prediction of whether the patient is in danger of AF during a sinus rhythm [101]. Recently, Sakli et al. [102] have presented an AI-based tool to classify 27 ECG features, and Elias et al. [103] have proposed a method to identify aortic stenosis, regurgitation, and mitral regurgitation in ECG. Implementation of AI-based ECG analysis does not only concern these cases. It has also helped to analyze if patients suffer from asymptomatic HF and to detect antiarrhythmic drugs and abnormal electrolyte levels, ventricular extrasystoles, atrial fibrillation, and left ventricular hypertrophy [104–108].

Antiplatelet therapy is important for cardiology patients who have undergone percutaneous coronary intervention (PCI). A population of 541 patients was studied to compare the effectiveness of treatment with ticagrelor or clopidogrel. Using a ML approach, the researchers found no difference in major adverse events, rehospitalization, or bleeding. However, ticagrelor showed better effects in patients with single-vessel disease [109].

Over 12,000 Caucasian patients were analyzed to determine the influence of aspirin intake on the prevalence of STEMI. Aspirin was connected with a decreased incidence of STEMI in patients with hypertension, hypercholesterolemia, and in smokers but not among patients with diabetes [110].

It is expected that atherosclerotic tissue presents different biomechanical properties than healthy tissue. An AI-based study by Karimi et al. [111] presented a model to biomechanically characterize atherosclerotic coronary arteries. Fuzzy logic was used to prepare a risk score for the onset of ischemic chronic leg ulcers in PAD patients and natural language processing to better diagnose PAD patients [112, 113]. AI methods have also been used among patients suffering from PAD to link them with potential limitations and symptom severity [114]. ML has been implemented to diagnose PAD based on gait analysis [115]. Age, diabetes mellitus and its complications, congestive HF, comorbidities, and earlier revascularisation are factors increasing an in-hospital mortality in PAD [116].

The aortic diameter might be connected with an occlusive vascular disease [117, 118]. Pirruccello et al. [119] presented GWAS of thoracic aorta describing 104 new loci and their association with aortic aneurysm or dissection. The study was performed on 39,688 individuals from a UK Biobank and is definitely a new direction in identifying asymptomatic patients at risk for an acute aortic syndrome.

Plasma lipids are a modifiable risk factor for CAD. Guo et al. [120] presented a novel marker—the atherogenic index of plasma (AIP)—that may become a novel predictor of CAD in Chinese postmenopausal women. Interestingly, the ILLUMINATE study of torcetrapib, a cholesterol ester transfer protein inhibitor, was closed after 550 days because of the increased rate of cardiovascular events (1.2%) and mortality (0.4%). Artificially created nanoparticles may be helpful in a new drug development [121]. The study of Williams et al. [122] was designed to analyze and explain the harmful mechanism of the drug and to determine whether it would have been possible to predict such outcomes earlier. Proteomics, the protein-based risk score, turned out to be a proper tool to predict the harm within 3 months. Benincasa et al. [123] proposed a digitalized way to individualize the treatment of dyslipidemia and Tsigalou et al. [124] presented a ML method to assess LDL plasma levels. Another study created a method to identify patients with familial hypercholesterolemia [125]. Interestingly, nondiabetic patients with chronic kidney disease may present a hidden proatherogenic lipid profile [126]. Stem cells play an important role in the pathogenesis of atherosclerosis. Their release into the bloodstream during acute myocardial infarction results in atherosclerosis progression. Li et al. [127] designed Atherosclerosis-risk Modules to better understand the pathophysiology of atherosclerosis from the perspective of the system's biology. Connecting AI, gene expression and human networks (signaling and inflammatory pathways) derived valuable information from a stem cell point of view. Biological networks were also investigated by other authors [128, 129]. Dan–Shen–Yin (DSY), a traditional Chinese formula comprising Salvia Miltrorrhiza, Fructus Amomi, and sandalwood, is broadly used in diabetes and CAD; however, the mechanism of action remains unknown. The study proposed integration of biology, proteomics, and experimental pharmacology to understand its influence on atherosclerosis [128]. Molecular understanding of pathophysiological pathways and genes with bioinformatics was performed in other studies as well [130–133]. They can be also used to identify new biomarkers for atherosclerosis [134–138], biomarkers connected with a particular ischemic stroke type [139], and determine if the plaque is rupture-prone [140]. Serum markers for diabetes, CAD, and diabetes associated with CAD were studied using AI as well [141]. The topic of AI in pediatric cardiology has also been raised [142, 143].

The role of the opportunistic imaging concept has also been raised in the literature. Examinations of knee MRI of osteoarthritis patients [144] and standardized knee MRI [145] were a focus of a study of atherosclerosis development within the popliteal artery using ML. AI-based studies which investigated plaque distribution and composition predicted the plaque progression [146, 147].  Table 4 presents studies that are included in this analysis.

## 6. Discussion

Precision phenomapping and ML will constantly gain in popularity. Crosstalk between various “omic” fields shows new paths that may be helpful in better understanding and treating CVDs. The multiomic approach generates big data impossible to analyze without AI solutions as most genetic studies are being conducted with combined methods, using software and other programs incorporating AI. Big data has been called the greatest untapped resource of mankind [85]. AI-based algorithms have made a substantial impact in better understanding of atherosclerosis, genetics, diagnosing CAD, and cardiovascular imaging. Some of them are descriptive studies that create a problem of repeatability of what was already mentioned above.

These new omic fields have been developed to better understand the genomic causes of atherosclerosis. New genes (inherited and de novo mutations) are still being discovered. Similarly, the extraction of radiomic features based on CT or MRI images to build AI-based systems dedicated to speeding up the workflow and providing accurate diagnosis is of paramount importance. Other analyses related to lipidology, PAD, drug discovery, and their interactions are included in the multiomic fields. Attempts are being made to overcome the problem of the black box phenomenon. Other ethical issues such as the “human factor” or the subjectivity and experience of a physician are currently being discussed. Will AI take over human tasks? These are the questions that have been raised, and there is still no proper and unequivocal answer. A simplified schema of intelligent data processing is presented in Figure 3.

## 7. Limitations

In the era of big data, special measures are required. There are also questions of boundaries with other areas, not strictly classified as AI and presented in this review. Some reviews concerning AI solutions implemented in the cardiovascular system are available [42, 46, 53]. However, the authors of this work aimed to present a broader point of view and included studies implementing AI in data analysis. For example, Depuydt et al. [15] presented big data analysis with the R 3.5 environment and Seurat 3.0 [15, 33]. “R” is a free software for statistical analysis and graphics and the R method is widely used in new-style AI, involving ML. Seurat uses ML for cell classification. Also, other studies implement SPSS [94, 110], PLINK [31, 38, 41, 42], CARDIoGRAMplusC4D [26, 34, 37], or Ingenuity [20, 23, 112] that are strictly correlated with AI. The search biases are unavoidable as well and the authors are aware of this. Moreover, the topic is extensive so the decision was made to exclude papers concerning an AI-based cardiovascular risk stratification as this will be given in another article. Also, the implementation of AI in PAD could be discussed more broadly [164]. Recently, an article raising a topic of AI in atherosclerosis has been published [165]. The article above however, discusses the problem more exhaustively, has been carefully planned and additionally focuses on precision medicine. Other articles present an insight into AI itself [166–170], discuss an application of a “Digital Twin” [171, 172] or an AI-application in various medical fields like nuclear medicine [173], genetics of CVDs [174], cardio-oncology [175–178], oncology [179], electrophysiology [180], assessment of a valvular heart disease [181], chronic diseases [182], and Alzheimer's [183]. This review was not reported and has no official protocol.

## 8. Conclusions

Personalized diagnostics and therapy have already changed the way we practice medicine. The potential of applying AI to the already overburdened healthcare system, with ever-increasing amounts of big data, seems inevitable. This article shows that the application of AI solutions in the light of the 4th industrial revolution has already begun. However, many complications need to be overcome. Not only cardiovascular risk stratification but also therapy and reduced time to diagnosis have become the benchmark in the diagnosis and treatment of atherosclerosis. This branch is still being developed.

## Figures and Tables

**Figure 1:** Identification of studies search: (1) “artificial intelligence” OR “AI” AND “atherosclerosis” (last 10 years) *n* = 4,458; (2) “artificial intelligence” OR “AI” AND “atherosclerosis” AND “cardiology” AND “GWAS” *n* = 110; (3) “artificial intelligence” OR “AI” AND “cardiology” AND “precision medicine” *n* = 352; and (4) “artificial intelligence” OR “AI” AND “cardiology” AND “radiomics” *n* = 31.

**Figure 2:** Artificial intelligence and its application in medical context.

**Figure 3:** Simplified schema of intelligent data processing.

**Table 1:** Methodology.

Criteria	Objectives
Inclusion criteria	Presence of AI solutions
	Application in personalized medicine

Exclusion criteria	Studies performed on animals
	Studies concerning cardiovascular risk stratification
	Verification of the methods impossible

Classification of articles	GWAS
	Radiomics
	Other studies
	Cardiovascular risk stratification (will be given in another article)

**Table 2:** Studies included in the GWAS-section analysis and AI methods applied.

References	Method of data analysis	AI approaches
Musunuru et al. [10]	SPSS	Machine learning
Shi et al. [11]	HAPGEN	Transfer learning
Li et al. [12]	STAAR	Machine learning
Piechotta et al. [13]	JACUSA	Machine learning
Yazdani et al. [14]	—	Bayesian causal network
Depuydt et al. [15]	Custom R scripts, Seurat	Machine learning
Örd et al. [17]	HOMER	Support vector regression
Aavik et al. [20]	Ingenuity	Machine learning
Folkersen et al. [21]	PLINK	Machine learning
Plens-Galaska [22]	GraphPad Prism	Machine learning
Pérez-Sánchez [23]	Ingenuity	Machine learning
Liu et al. [24]	R package	Machine learning
Zekavat et al. [35]	WGS, logistic regression	Machine learning
Nelson et al. [26]	CARDIoGRAMplusC4D	Machine learning
Manichaikul et al. [28]	SMARTPCA, KING	Machine learning
Aherrahrou et al. [30]	GraphPad Prism	Machine learning
Aherrahrou et al. [31]	PLINK, R package, GraphPad Prism	Machine learning
Meng et al. [32]	R package, Cytoscape	Machine learning
Karjalainen et al. [34]	CARDIoGRAMplusC4D	Machine learning
Richardson et al. [37]	CARDIoGRAMplusC4D	Machine learning
Hoekstra et al. [36]	PLINK	Machine learning
Holliday et al. [38]	PLINK, METAL	Machine learning
Awan et al. [39]	R package, MCODE	Machine learning
Lu et al. [40]	LDhat package, METAL	Machine learning
Shendre et al. [41]	LAMPLD, PLINK	Machine learning
Shrestha et al. [42]	PLINK	Machine learning

**Table 3:** Studies included in the radiomics-section analysis and AI methods applied.

References	Method of data analysis	AI approaches
Huang et al. [44]	—	Convolutional neural networks
Sanchez-Martinez et al. [46]	—	Machine learning, clustering
Madani et al. [47]	—	Convolutional neural networks
Soto et al. [48]	—	Deep learning
Duffy et al. [49]	—	Deep learning
Yuan et al. [50]	—	Deep learning
Liu et al. [51]	—	Deep learning
Kay et al. [54]	—	Machine learning, logistic regression
Hu et al. [60]	—	Logistic regression
Gupta et al. [61]	—	Deep neural network
Atkov et al. [62]	—	Deep neural network
Lin et al. [64]	—	Machine learning
Coenen et al. [65]	—	Machine learning
Al'Aref et al. [66]	—	Machine learning
von Knebel Doeberitz et al. [68]	—	Deep learning
Lee et al. [70]	—	Machine learning
Bajaj et al. [71]	—	Machine learning
Amato et al. [72]	—	Unsupervised machine learning
Oikonomou et al. [74]	—	Machine learning
Commandeur et al. [75]	—	Deep learning
Eisenberg [76]	—	Deep learning
Chen et al. [78]	—	Unsupervised machine learning
Wu et al. [79]	—	Deep neural networks
Antonopoulos et al. [80]	—	Machine learning
Sengupta et al. [81]	—	Machine learning
Sparapani et al. [82]	—	Bayesian additive regression trees
Ma et al. [83]	—	Machine learning
Durmaz et al. [84]	—	Machine learning
Laudicella et al. [86]	—	Deep neural networks
Nakajima et al. [87]	—	Deep neural networks
Hu et al. [88]	—	Machine learning
Betancur et al. [89]	—	Deep learning
Betancur et al. [90]	—	Machine learning
Arsanjani et al. [92]	—	Machine learning
Lin et al. [93]	—	Machine learning
Baumann et al. [94]	—	Machine learning
Suinesiaputra et al. [95]	—	Deep neural networks
Lossnitzer et al. [96]	—	Machine learning
Lossnitzer et al. [97]	—	Machine learning
Lee et al. [70]	SPSS	Machine learning (binary class L2 penalized logistic regression, deep neural networks, random forest, AdaBoost, CatBoost, and support vector machine)
Ji et al. [98]	SPSS	Deep learning

**Table 4:** Studies included in the other studies-section analysis and AI methods applied.

References	Method of data analysis	AI approaches
Zhao et al. [99]	—	Deep neural networks
Makimoto et al. [100]	SPSS	Deep neural networks
Attia et al. [101]	—	Deep neural networks
Sakli et al. [102]	—	Deep neural networks
Elias et al. [103]	—	Deep neural networks
Sangha et al. [105]	—	Deep neural networks
Chang et al. [106]	—	Deep neural networks
Liu et al. [107]	—	Machine learning (decision tree, K-means, back propagation neural network)
Tutuko et al. [108]	—	Deep neural networks
Xue et al. [109]	—	Decision tree
Burgiardini et al. [110]	SPSS	Supervised machine learning (k nearest neighbor algorithm)
Karimi et al. [111]	—	Deep neural networks
Serra et al. [112]	—	Fuzzy logic
Weissler et al. [113]	—	Natural language processing
Baloch et al. [114]	—	Supervised machine learning
Al Ramini et al. [115]	—	Machine learning
Zhang et al. [116]	—	Machine learning
Laughlin et al. [117]	SPSS	Machine learning
Pirruccello et al. [119]	—	Deep learning
Guo et al. [120]	SPSS	Machine learning
Williams et al. [122]	Ingenuity	Machine learning
Tsigalou et al. [124]	—	Machine learning
Paragh et al. [125]	—	Deep neural networks (natural language processing- word2vec)
Bermudez-Lopez et al. [126]	—	Machine learning (random forest analysis)
Li et al. [127]	—	Human signaling networks, ClusterONE
Yang et al. [128]	Cytoscape, MCODE	Machine learning
Wang et al. [129]	DAVID, SPSS	Machine learning
Tan et al. [130]	Cytoscape, MCODE	Machine learning
Zhang et al. [131]	Cytoscape, MCODE	Machine learning
Nai et al. [132]	Cytoscape, R package	Machine learning
Huang et al. [134]	Cytoscape	Machine learning
Yagi et al. [135]	GeneSpring	Machine learning
Liu et al. [136]	Cluster 3.0 genes, Python	Machine learning
Johno et al. [137]	—	Machine learning
Wei and Quan [138]	DAVID	Machine learning
Wang et al. [139]	Clustering, DAVID, Cytoscape, MCODE	Machine learning
Wang et al. [140]	DAVID, R package, Cytoscape, MCODE	Machine learning
Adela et al. [141]	—	Random forest analysis
Canton et al. [144]	—	Deep neural networks
Chen et al. [145]	—	Deep neural networks
Jurtz et al. [146]	—	Deep learning
Kigka et al. [147]	—	Machine learning
Wang et al. [148]	—	Machine learning
Xu et al. [149]	—	Machine learning
Forrest et al. [150]	—	Machine learning
Yang et al. [151]	—	Machine learning
Sharma et al. [152]	—	Machine learning
Chen et al. [153]	—	Machine learning
Jones et al. [154]	—	Machine learning
Jiang et al. [155]	—	Machine learning
Ross et al. [156]	—	Machine learning
Fan et al. [157]	—	Machine learning
Cox et al. [158]	—	Machine learning
Gao et al. [159]	—	Machine learning (logistic regression, random forest)
Kumar and Priya [160]	—	Machine learning (support vector machine, kernel radial basis function)
Park et al. [161]	—	Machine learning
Dai et al. [162]	—	Supervised convolutional neural network
Afzal et al. [163]	—	Natural language processing

## Data Availability

No new data were created or analyzed in this study. Data sharing is not applicable to this article.

## References

[1] Freeth T., Bitsakis Y., Moussas X. (2006). Decoding the ancient greek astronomical calculator known as the antikythera mechanism. *Nature*.

[2] Kool L., Dekker F., Bunschoten A. (2020). Gold and silver dichroic nanocomposite in the quest for 3D printing the Lycurgus cup. *Beilstein Journal of Nanotechnology*.

[3] Kirkby M. J. (1983). The fractal geometry of nature. Benoit B. Mandelbrot. W. H. Freeman and co., San Francisco, 1982. No. of pages: 460. Price: £22.75 (hardback). *Earth Surface Processes and Landforms*.

[4] Metze K., Adam R., Florindo J. B. (2019). The fractal dimension of chromatin—a potential molecular marker for carcinogenesis, tumor progression and prognosis. *Expert Review of Molecular Diagnostics*.

[5] Bartkiewicz K., Gneiting C., Černoch A., Jiráková K., Lemr K., Nori F. (2020). Experimental kernel-based quantum machine learning in finite feature space. *Scientific Reports*.

[6] Herrington W., Lacey B., Sherliker P., Armitage J., Lewington S. (2016). Epidemiology of atherosclerosis and the potential to reduce the global burden of atherothrombotic disease. *Circulation Research*.

[7] Boyle E. A., Li Y. I., Pritchard J. K. (2017). An expanded view of complex traits: from polygenic to omnigenic. *Cell*.

[8] Lorkowski J., Kolaszyńska O., Pokorski M. (2021). Artificial intelligence and precision medicine: a perspective. *Integrative Clinical Research*.

[9] Hamamoto R., Komatsu M., Takasawa K., Asada K., Kaneko S. (2020). Epigenetics analysis and integrated analysis of multiomics data, including epigenetic data, using artificial intelligence in the era of precision medicine. *Biomolecules*.

[10] Musunuru K., Strong A., Frank-Kamenetsky M. (2010). From noncoding variant to phenotype via SORT1 at the 1p13 cholesterol locus. *Nature*.

[11] Shi H., Kichaev G., Pasaniuc B. (2016). Contrasting the genetic architecture of 30 complex traits from summary association data. *The American Journal of Human Genetics*.

[12] Li X., Li Z., Zhou H. (2020). Dynamic incorporation of multiple in silico functional annotations empowers rare variant association analysis of large whole-genome sequencing studies at scale. *Nature Genetics*.

[13] Piechotta M., Wyler E., Ohler U., Landthaler M., Dieterich C. (2017). JACUSA: site-specific identification of RNA editing events from replicate sequencing data. *BMC Bioinformatics*.

[14] Yazdani A., Mendez-Giraldez R., Yazdani A., Kosorok M. R., Roussos P. (2020). Differential gene regulatory pattern in the human brain from schizophrenia using transcriptomic-causal network. *BMC Bioinformatics*.

[15] Depuydt M. A. C., Prange K. H. M., Slenders L. (2020). Microanatomy of the human atherosclerotic plaque by single-cell transcriptomics. *Circulation Research*.

[16] Willemsen L., de Winther M. P. J. (2020). Macrophage subsets in atherosclerosis as defined by single-cell technologies. *The Journal of Pathology*.

[17] Örd T., Õunap K., Stolze L. K. (2021). Single-cell epigenomics and functional fine-mapping of atherosclerosis GWAS loci. *Circulation Research*.

[18] Jin L., Hong N., Ai X. (2021). LncRNAs as therapeutic targets for autophagy-involved cardiovascular diseases: a review of molecular mechanism and therapy strategy. *Current Medicinal Chemistry*.

[19] Poller W., Dimmeler S., Heymans S. (2018). Non-coding RNAs in cardiovascular diseases: diagnostic and therapeutic perspectives. *European Heart Journal*.

[20] Aavik E., Lumivuori H., Leppanen O. (2015). Global DNA methylation analysis of human atherosclerotic plaques reveals extensive genomic hypomethylation and reactivation at imprinted locus 14q32 involving induction of a miRNA cluster. *European Heart Journal*.

[21] Folkersen L., Gustafsson S., Wang Q. (2020). Genomic and drug target evaluation of 90 cardiovascular proteins in 30,931 individuals. *Nature Metabolism*.

[22] Plens-Galaska M., Szelag M., Collado A. (2018). Genome-wide inhibition of pro-atherogenic gene expression by multi-STAT targeting compounds as a novel treatment strategy of CVDs. *Frontiers in Immunology*.

[23] Pérez-Sánchez L., Patiño-Trives A. M., Aguirre-Zamorano M. Á. (2021). Characterization of antiphospholipid syndrome atherothrombotic risk by unsupervised integrated transcriptomic analyses. *Arteriosclerosis, Thrombosis, and Vascular Biology*.

[24] Liu W., Zhao Y., Wu J. (2018). Gene expression profile analysis of the progression of carotid atherosclerotic plaques. *Molecular Medicine Reports*.

[25] Erdmann J., Kessler T., Munoz Venegas L., Schunkert H. (2018). A decade of genome-wide association studies for coronary artery disease: the challenges ahead. *Cardiovascular Research*.

[26] EPIC-CVD Consortium, CARDIoGRAMplusC4D, The UK Biobank CardioMetabolic Consortium CHD working group (2017). Association analyses based on false discovery rate implicate new loci for coronary artery disease. *Nature Genetics*.

[27] Jadhav K. S., Bauer R. C. (2019). Trouble with tribbles-1. *Arteriosclerosis, Thrombosis, and Vascular Biology*.

[28] Manichaikul A., Palmas W., Rodriguez C. J. (2012). Population structure of Hispanics in the United States: the multi-ethnic study of atherosclerosis. *PLOS Genetics*.

[29] Hu K. Y., Bauer R. C. (2021). Competing tissue-specific functions for the tribbles-1 plasma lipid associated locus. *Current Opinion in Lipidology*.

[30] Aherrahrou R., Aherrahrou Z., Schunkert H., Erdmann J. (2017). Coronary artery disease associated gene Phactr1 modulates severity of vascular calcification in vitro. *Biochemical and Biophysical Research Communications*.

[31] Aherrahrou R., Guo L., Nagraj V. P. (2020). Genetic regulation of atherosclerosis-relevant phenotypes in human vascular smooth muscle cells. *Circulation Research*.

[32] Meng Y., Zhang C., Liang L. (2021). Identification of potential key genes involved in the carotid atherosclerosis. *Clinical Interventions in Aging*.

[33] Levin M. G., Klarin D., Assimes T. L. (2021). Genetics of smoking and risk of atherosclerotic cardiovascular diseases: a mendelian randomization study. *JAMA Network Open*.

[34] Karjalainen M. K., Holmes M. V., Wang Q. (2020). Apolipoprotein A-I concentrations and risk of coronary artery disease: a mendelian randomization study. *Atherosclerosis*.

[35] Zekavat S. M., Ruotsalainen S., Handsaker R. E. (2018). Deep coverage whole genome sequences and plasma lipoprotein(a) in individuals of European and African ancestries. *Nature Communications*.

[36] Hoekstra M., Chen H. Y., Rong J. (2021). Genome-wide association study highlights APOH as a novel locus for lipoprotein(a) levels-brief report. *Arteriosclerosis, Thrombosis, and Vascular Biology logo*.

[37] Richardson T. G., Sanderson E., Palmer T. M. (2020). Evaluating the relationship between circulating lipoprotein lipids and apolipoproteins with risk of coronary heart disease: a multivariable Mendelian randomisation analysis. *PLOS Medicine*.

[38] Holliday E. G., Traylor M., Malik R. (2015). Genetic overlap between diagnostic subtypes of ischemic stroke. *Stroke*.

[39] Awan Z., Alrayes N., Khan Z. (2022). Identifying significant genes and functionally enriched pathways in familial hypercholesterolemia using integrated gene co-expression network analysis. *Saudi Journal of Biological Sciences*.

[40] Lu Y., Dimitrov L., Chen S.-H. (2021). Multiethnic genome-wide association study of subclinical atherosclerosis in individuals with type 2 diabetes. *Circulation: Genomic and Precision Medicine*.

[41] Shendre A., Wiener H. W., Irvin M. R. (2017). Genome-wide admixture and association study of subclinical atherosclerosis in the Women’s Interagency HIV Study (WIHS). *PLOS ONE*.

[42] Shrestha S., Irvin M. R., Taylor K. D. (2010). A genome-wide association study of carotid atherosclerosis in HIV-infected men. *AIDS*.

[43] Seetharam K., Brito D., Farjo P. D., Sengupta P. P. (2020). The role of artificial intelligence in cardiovascular imaging: state of the art review. *Frontiers in Cardiovascular Medicine*.

[44] Huang K.-C., Huang C.-S., Su M.-Y. (2021). Artificial intelligence aids cardiac image quality assessment for improving precision in strain measurements. *JACC: Cardiovascular Imaging*.

[45] Ahmad F. S., Luo Y., Wehbe R. M., Thomas J. D., Shah S. J. (2022). Advances in machine learning approaches to heart failure with preserved ejection fraction. *Heart Failure Clinics*.

[46] Sanchez-Martinez S., Duchateau N., Erdei T. (2018). Machine learning analysis of left ventricular function to characterize heart failure with preserved ejection fraction. *Circulation: Cardiovascular Imaging*.

[47] Madani A., Arnaout R., Mofrad M., Arnaout R. (2018). Fast and accurate view classification of echocardiograms using deep learning. *NPJ Digital Medicine*.

[48] Soto J. T., Hughes J. W., Sanchez P. A., Perez M., Ouyang D., Ashley E. A. (2022). Multimodal deep learning enhances diagnostic precision in left ventricular hypertrophy. *European Heart Journal-Digital Health*.

[49] Duffy G., Cheng P. P., Yuan N. (2022). High-throughput precision phenotyping of left ventricular hypertrophy with cardiovascular deep learning. *JAMA Cardiology*.

[50] Yuan N., Kwan A. C., Duffy G. (2022). Prediction of coronary artery calcium using deep learning of echocardiograms. *Journal of the American Society of Echocardiography*.

[51] Liu B., Chang H., Yang D. (2023). A deep learning framework assisted echocardiography with diagnosis, lesion localization, phenogrouping heterogeneous disease, and anomaly detection. *Scientific Reports*.

[52] Mathur P., Srivastava S., Xu X., Mehta J. L. (2020). Artificial intelligence, machine learning, and cardiovascular disease. *Clinical Medicine Insights: Cardiology*.

[53] Al’Aref S. J., Anchouche K., Singh G. (2019). Clinical applications of machine learning in cardiovascular disease and its relevance to cardiac imaging. *European Heart Journal*.

[54] Kay F. U., Abbara S., Joshi P. H., Garg S., Khera A., Peshock R. M. (2020). Identification of high-risk left ventricular hypertrophy on calcium scoring cardiac computed tomography scans: validation in the DHS. *Circulation: Cardiovascular Imaging*.

[55] Nicol E. D., Norgaard B. L., Blanke P. (2019). The future of cardiovascular computed tomography. *JACC: Cardiovascular Imaging*.

[56] Alharbi Y., Otton J., Muller D. W. M. (2020). Predicting the outcome of transcatheter mitral valve implantation using image-based computational models. *Journal of Cardiovascular Computed Tomography*.

[57] Yuan X., Kan X., Xu X. Y., Nienaber C. A. (2020). Finite element modeling to predict procedural success of thoracic endovascular aortic repair in type A aortic dissection. *JTCVS Techniques*.

[58] Jia D., Jeon B., Park H.-B., Chang H.-J., Zhang L. T. (2019). Image-based flow simulations of pre- and post-left atrial appendage closure in the left atrium. *Cardiovascular Engineering and Technology*.

[59] Bosi G. M., Capelli C., Cheang M. H. (2018). Population-specific material properties of the implantation site for transcatheter aortic valve replacement finite element simulations. *Journal of Biomechanics*.

[60] Hu W., Wu X., Dong D. (2020). Novel radiomics features from CCTA images for the functional evaluation of significant ischaemic lesions based on the coronary fractional flow reserve score. *The International Journal of Cardiovascular Imaging*.

[61] Gupta V., Demirer M., Bigelow M. (2020). Performance of a deep neural network algorithm based on a small medical image dataset: incremental impact of 3D-to-2D reformation combined with novel data augmentation, photometric conversion, or transfer learning. *Journal of Digital Imaging*.

[62] Atkov O. Y., Gorokhova S. G., Sboev A. G. (2012). Coronary heart disease diagnosis by artificial neural networks including genetic polymorphisms and clinical parameters. *Journal of Cardiology*.

[63] Dey D., Slomka P. J., Leeson P. (2019). Artificial intelligence in cardiovascular imaging. *Journal of the American College of Cardiology*.

[64] Lin A., Kolossváry M., Cadet S. (2022). Radiomics-based precision phenotyping identifies unstable coronary plaques from computed tomography angiography. *JACC: Cardiovascular Imaging*.

[65] Coenen A., Kim Y.-H., Kruk M. (2018). Diagnostic accuracy of a machine-learning approach to coronary computed tomographic angiography-based fractional flow reserve. *Circulation: Cardiovascular Imaging*.

[66] Al’Aref S. J., Maliakal G., Singh G. (2020). Machine learning of clinical variables and coronary artery calcium scoring for the prediction of obstructive coronary artery disease on coronary computed tomography angiography: analysis from the CONFIRM registry. *European Heart Journal*.

[67] Cau R., Flanders A., Mannelli L. (2021). Artificial intelligence in computed tomography plaque characterization: a review. *European Journal of Radiology*.

[68] von Knebel Doeberitz P. L., De Cecco C. N., Schoepf U. J. (2019). Coronary CT angiography-derived plaque quantification with artificial intelligence CT fractional flow reserve for the identification of lesion-specific ischemia. *European Radiology*.

[69] Oikonomou E. K., Siddique M., Antoniades C. (2020). Artificial intelligence in medical imaging: a radiomic guide to precision phenotyping of cardiovascular disease. *Cardiovascular Research*.

[70] Lee J.-G., Ko J., Hae H. (2020). Intravascular ultrasound-based machine learning for predicting fractional flow reserve in intermediate coronary artery lesions. *Atherosclerosis*.

[71] Bajaj R., Eggermont J., Grainger S. J. (2022). Machine learning for atherosclerotic tissue component classification in combined near-infrared spectroscopy intravascular ultrasound imaging: validation against histology. *Atherosclerosis*.

[72] Amato M., Buscema M., Massini G. (2021). Assessment of new coronary features on quantitative coronary angiographic images with innovative unsupervised artificial adaptive systems: a proof-of-concept study. *Frontiers in Cardiovascular Medicine*.

[73] Bartelt A., Leipsic J., Weber C. (2019). The new age of radiomic risk profiling: perivascular fat at the heart of the matter. *European Heart Journal*.

[74] Oikonomou E. K., Williams M. C., Kotanidis C. P. (2019). A novel machine learning-derived radiotranscriptomic signature of perivascular fat improves cardiac risk prediction using coronary CT angiography. *European Heart Journal*.

[75] Commandeur F., Goeller M., Betancur J. (2018). Deep learning for quantification of epicardial and thoracic adipose tissue from non-contrast CT. *IEEE Transactions on Medical Imaging*.

[76] Eisenberg E., McElhinney P. A., Commandeur F. (2020). Deep learning–based quantification of epicardial adipose tissue volume and attenuation predicts major adverse cardiovascular events in asymptomatic subjects. *Circulation: Cardiovascular Imaging*.

[77] Ponikowski P., Voors A. A., Anker S. D. (2016). 2016 ESC Guidelines for the diagnosis and treatment of acute and chronic heart failure. *European Heart Journal*.

[78] Chen L., Zhao H., Jiang H. (2021). Domain adaptive and fully automated carotid artery atherosclerotic lesion detection using an artificial intelligence approach (LATTE) on 3D MRI. *Magnetic Resonance in Medicine*.

[79] Wu J., Xin J., Yang X. (2019). Deep morphology aided diagnosis network for segmentation of carotid artery vessel wall and diagnosis of carotid atherosclerosis on black-blood vessel wall MRI. *Medical Physics*.

[80] Antonopoulos A. S., Boutsikou M., Simantiris S. (2021). Machine learning of native T1 mapping radiomics for classification of hypertrophic cardiomyopathy phenotypes. *Scientific Reports*.

[81] Sengupta P. P., Shrestha S., Kagiyama N. (2021). A machine-learning framework to identify distinct phenotypes of aortic stenosis severity. *JACC: Cardiovascular Imaging*.

[82] Sparapani R., Dabbouseh N. M., Gutterman D. (2019). Detection of left ventricular hypertrophy using Bayesian additive regression trees: the MESA (multi-ethnic study of atherosclerosis). *Journal of the American Heart Association*.

[83] Ma Q., Ma Y., Yu T., Sun Z., Hou Y. (2021). Radiomics of non-contrast-enhanced T1 mapping: diagnostic and predictive performance for myocardial injury in acute ST-segment-elevation myocardial infarction. *Korean Journal of Radiology*.

[84] Durmaz E. S., Karabacak M., Ozkara B. B. (2023). Radiomics-based machine learning models in STEMI: a promising tool for the prediction of major adverse cardiac events. *European Radiology*.

[85] Lorkowski J., Grzegorowska O., Pokorski M. (2021). Artificial intelligence in the healthcare system: an overview. *Yeast Membrane Transport*.

[86] Laudicella R., Comelli A., Stefano A. (2021). Artificial neural networks in cardiovascular diseases and its potential for clinical application in molecular imaging. *Current Radiopharmaceuticals*.

[87] Nakajima K., Okuda K., Watanabe S. (2018). Artificial neural network retrained to detect myocardial ischemia using a Japanese multicenter database. *Annals of Nuclear Medicine*.

[88] Hu L.-H., Betancur J., Sharir T. (2020). Machine learning predicts per-vessel early coronary revascularization after fast myocardial perfusion SPECT: results from multicentre REFINE SPECT registry. *European Heart Journal-Cardiovascular Imaging*.

[89] Betancur J., Hu L.-H., Commandeur F. (2019). Deep learning analysis of upright-supine high-efficiency SPECT myocardial perfusion imaging for prediction of obstructive coronary artery disease: a multicenter study. *Journal of Nuclear Medicine*.

[90] Betancur J., Rubeaux M., Fuchs T. A. (2017). Automatic valve plane localization in myocardial perfusion SPECT/CT by machine learning: anatomic and clinical validation. *Journal of Nuclear Medicine*.

[91] Sollini M., Bandera F., Kirienko M. (2019). Quantitative imaging biomarkers in nuclear medicine: from SUV to image mining studies. Highlights from annals of nuclear medicine 2018. *European Journal of Nuclear Medicine and Molecular Imaging*.

[92] Arsanjani R., Xu Y., Dey D. (2013). Improved accuracy of myocardial perfusion SPECT for detection of coronary artery disease by machine learning in a large population. *Journal of Nuclear Cardiology*.

[93] Lin A., van Diemen P. A., Motwani M. (2022). Machine learning from quantitative coronary computed tomography angiography predicts fractional flow reserve-defined ischemia and impaired myocardial blood flow. *Circulation: Cardiovascular Imaging*.

[94] Baumann S., Hirt M., Rott C. (2020). Comparison of machine learning computed tomography-based fractional flow reserve and coronary CT angiography-derived plaque characteristics with invasive resting full-cycle ratio. *Journal of Clinical Medicine*.

[95] Suinesiaputra A., Mauger C. A., Ambale-Venkatesh B. (2022). Deep learning analysis of cardiac MRI in legacy datasets: multi-ethnic study of atherosclerosis. *Frontiers in Cardiovascular Medicine*.

[96] Lossnitzer D., Klenantz S., Andre F. (2022). Stable patients with suspected myocardial ischemia: comparison of machine-learning computed tomography-based fractional flow reserve and stress perfusion cardiovascular magnetic resonance imaging to detect myocardial ischemia. *BMC Cardiovascular Disorders*.

[97] Lossnitzer D., Chandra L., Rutsch M. (2020). Additional value of machine-learning computed tomographic angiography-based fractional flow reserve compared to standard computed tomographic angiography. *Journal of Clinical Medicine*.

[98] Ji F., Zhou S., Bi Z. (2021). Computed tomography angiography under deep learning in the treatment of atherosclerosis with rapamycin. *Journal of Healthcare Engineering*.

[99] Zhao Y., Xiong J., Hou Y. (2020). Early detection of ST-segment elevated myocardial infarction by artificial intelligence with 12-lead electrocardiogram. *International Journal of Cardiology*.

[100] Makimoto H., Höckmann M., Lin T. (2020). Performance of a convolutional neural network derived from an ECG database in recognizing myocardial infarction. *Scientific Reports*.

[101] Attia Z. I., Noseworthy P. A., Lopez-Jimenez F. (2019). An artificial intelligence-enabled ECG algorithm for the identification of patients with atrial fibrillation during sinus rhythm: a retrospective analysis of outcome prediction. *The Lancet*.

[102] Sakli N., Ghabri H., Soufiene B. O. (2022). ResNet-50 for 12-lead electrocardiogram automated diagnosis. *Computational Intelligence and Neuroscience*.

[103] Elias P., Poterucha T. J., Rajaram V. (2022). Deep learning electrocardiographic analysis for detection of left-sided valvular heart disease. *Journal of The American College of Cardiology*.

[104] Anderson K. P. (2019). Artificial intelligence-augmented ECG assessment: the promise and the challenge. *Journal of Cardiovascular Electrophysiology*.

[105] Sangha V., Mortazavi B. J., Haimovich A. D. (2022). Automated multilabel diagnosis on electrocardiographic images and signals. *Nature Communications*.

[106] Chang S.-N., Tseng Y.-H., Chen J.-J. (2022). An artificial intelligence-enabled ECG algorithm for identifying ventricular premature contraction during sinus rhythm. *European Journal of Medical Research*.

[107] Liu C.-W., Wu F.-H., Hu Y.-L. (2023). Left ventricular hypertrophy detection using electrocardiographic signal. *Scientific Reports*.

[108] Tutuko B., Rachmatullah M. N., Darmawahyuni A. (2022). Short single-lead ECG signal delineation-based deep learning: implementation in automatic atrial fibrillation identification. *Sensors*.

[109] Xue Y., Hu Z., Jing Y. (2020). Efficacy assessment of ticagrelor versus clopidogrel in Chinese patients with acute coronary syndrome undergoing percutaneous coronary intervention by data mining and machine-learning decision tree approaches. *Journal of Clinical Pharmacy and Therapeutics*.

[110] Bugiardini R., Pavasović S., Yoon J. (2020). Aspirin for primary prevention of ST segment elevation myocardial infarction in persons with diabetes and multiple risk factors. *eClinicalMedicine*.

[111] Karimi A., Rahmati S. M., Sera T., Kudo S., Navidbakhsh M. (2017). A combination of constitutive damage model and artificial neural networks to characterize the mechanical properties of the healthy and atherosclerotic human coronary arteries. *Artificial Organs*.

[112] Serra R., Bracale U. M., Barbetta A. (2020). PredyCLU: a prediction system for chronic leg ulcers based on fuzzy logic; part II—exploring the arterial side. *International Wound Journal*.

[113] Weissler E. H., Zhang J., Lippmann S., Rusincovitch S., Henao R., Jones W. S. (2020). Use of natural language processing to improve identification of patients with peripheral artery disease. *Circulation: Cardiovascular Interventions*.

[114] Qutrio Baloch Z., Raza S. A., Pathak R., Marone L., Ali A. (2020). Machine learning confirms nonlinear relationship between severity of peripheral arterial disease, functional limitation and symptom severity. *Diagnostics*.

[115] Al-Ramini A., Hassan M., Fallahtafti F. (2022). Machine learning-based peripheral artery disease identification using laboratory-based gait data. *Sensors*.

[116] Zhang D., Li Y., Kalbaugh C. A. (2022). Machine learning approach to predict in-hospital mortality in patients admitted for peripheral artery disease in the United States. *Journal of the American Heart Association*.

[117] Laughlin G. A., Allison M. A., Jensky N. E. (2011). Abdominal aortic diameter and vascular atherosclerosis: the multi-ethnic study of atherosclerosis. *European Journal of Vascular and Endovascular Surgery*.

[118] Genkel V., Kuznetcova A., Shaposhnik I. (2021). Relationship between the abdominal aortic diameter and carotid atherosclerosis in middle-aged patients without established atherosclerotic cardiovascular diseases. *International Angiology*.

[119] Pirruccello J. P., Chaffin M. D., Chou E. L. (2022). Deep learning enables genetic analysis of the human thoracic aorta. *Nature Genetics*.

[120] Guo Q., Zhou S., Feng X. (2020). The sensibility of the new blood lipid indicator—atherogenic index of plasma (AIP) in menopausal women with coronary artery disease. *Lipids in Health and Disease*.

[121] Kornmueller K., Vidakovic I., Prassl R. (2019). Artificial high density lipoprotein nanoparticles in cardiovascular research. *Molecules*.

[122] Williams S. A., Murthy A. C., DeLisle R. K. (2018). Improving assessment of drug safety through proteomics: early detection and mechanistic characterization of the unforeseen harmful effects of torcetrapib. *Circulation*.

[123] Benincasa G., de Candia P., Costa D. (2021). Network medicine approach in prevention and personalized treatment of dyslipidemias. *Lipids*.

[124] Tsigalou C., Panopoulou M., Papadopoulos C., Karvelas A., Tsairidis D., Anagnostopoulos K. (2021). Estimation of low-density lipoprotein cholesterol by machine learning methods. *Clinica Chimica Acta*.

[125] Paragh G., Harangi M., Karányi Z., Daróczy B., Németh Á., Fülöp P. (2018). Identifying patients with familial hypercholesterolemia using data mining methods in the northern great plain region of Hungary. *Atherosclerosis*.

[126] Bermudez-Lopez M., Forne C., Amigo N. (2019). An in-depth analysis shows a hidden atherogenic lipoprotein profile in non-diabetic chronic kidney disease patients. *Expert Opinion on Therapeutic Targets*.

[127] Li W., Huang H., Li L. (2018). The pathogenesis of atherosclerosis based on human signaling networks and stem cell expression data. *International Journal of Biological Sciences*.

[128] Yang K., Zeng L., Ge A. (2020). Integrating systematic biological and proteomics strategies to explore the pharmacological mechanism of danshen yin modified on atherosclerosis. *Journal of Cellular and Molecular Medicine*.

[129] Wang D., Tian L., Shi C. (2020). Network pharmacology-based prediction of the active ingredients and mechanism of Shen Gui capsule for application to coronary heart disease. *Computers in Biology and Medicine*.

[130] Tan X., Zhang X., Pan L., Tian X., Dong P. (2017). Identification of key pathways and genes in advanced coronary atherosclerosis using bioinformatics analysis. *BioMed Research International*.

[131] Zhang Y.-M., Meng L.-B., Yu S.-J., Ma D.-X. (2020). Identification of potential crucial genes in monocytes for atherosclerosis using bioinformatics analysis. *Journal of International Medical Research*.

[132] Nai W., Threapleton D., Lu J. (2016). Identification of novel genes and pathways in carotid atheroma using integrated bioinformatic methods. *Scientific Reports*.

[133] Zawada A. M., Rogacev K. S., Müllerm S. (2014). Massive analysis of cDNA Ends (MACE) and miRNA expression profiling identifies proatherogenic pathways in chronic kidney disease. *Epigenetics*.

[134] Huang H.-M., Jiang X., Hao M.-L. (2019). Identification of biomarkers in macrophages of atherosclerosis by microarray analysis. *Lipids in Health and Disease*.

[135] Yagi H., Nishigori M., Murakami Y. (2020). Discovery of novel biomarkers for atherosclerotic aortic aneurysm through proteomics-based assessment of disease progression. *Scientific Reports*.

[136] Liu L., Liu Y., Liu C., Zhang Z., Du Y., Zhao H. (2016). Analysis of gene expression profile identifies potential biomarkers for atherosclerosis. *Molecular Medicine Reports*.

[137] Johno H., Yoshimura K., Mori Y. (2018). Detection of potential new biomarkers of atherosclerosis by probe electrospray ionization mass spectrometry. *Metabolomics*.

[138] Wei L. K., Quan L. S. (2019). Biomarkers for ischemic stroke subtypes: a protein–protein interaction analysis. *Computational Biology and Chemistry*.

[139] Wang W., Zhang K., Zhang H. (2019). Underlying genes involved in atherosclerotic macrophages: insights from microarray data mining. *Medical Science Monitor*.

[140] Wang H., Liu D., Zhang H. (2019). Investigation of the underlying genes and mechanism of macrophage-enriched ruptured atherosclerotic plaques using bioinformatics method. *Journal of Atherosclerosis and Thrombosis*.

[141] Adela R., Reddy P. N. C., Ghosh T. S. (2019). Serum protein signature of coronary artery disease in type 2 diabetes mellitus. *Journal of Translational Medicine*.

[142] Gaffar S., Gearhart A. S., Chang A. C. (2020). The next frontier in pediatric cardiology: artificial intelligence. *Pediatric Clinics of North America*.

[143] Sethi Y., Patel N., Kaka N. (2022). Artificial intelligence in pediatric cardiology: a scoping review. *Journal of Clinical Medicine*.

[144] Canton G., Hippe D. S., Chen L. (2021). Atherosclerotic burden and remodeling patterns of the popliteal artery as detected in the magnetic resonance imaging osteoarthritis initiative data set. *Journal of the American Heart Association*.

[145] Chen L., Canton G., Liu W. (2020). Fully automated and robust analysis technique for popliteal artery vessel wall evaluation (FRAPPE) using neural network models from standardized knee MRI. *Magnetic Resonance in Medicine*.

[146] Jurtz V. I., Skovbjerg G., Salinas C. G. (2020). Deep learning reveals 3D atherosclerotic plaque distribution and composition. *Scientific Reports*.

[147] Kigka V. I., Sakellarios A. I., Tsompou P. Site specific prediction of atherosclerotic plaque progression using computational biomechanics and machine learning.

[148] Wang J., Kang Z., Liu Y., Li Z., Liu Y., Liu J. (2022). Identification of immune cell infiltration and diagnostic biomarkers in unstable atherosclerotic plaques by integrated bioinformatics analysis and machine learning. *Frontiers in Immunology*.

[149] Xu J., Zhou H., Cheng Y., Xiang G. (2022). Identifying potential signatures for atherosclerosis in the context of predictive, preventive, and personalized medicine using integrative bioinformatics approaches and machine-learning strategies. *EPMA Journal*.

[150] Forrest I. S., Petrazzini B. O., Duffy Á. (2023). Machine learning-based marker for coronary artery disease: derivation and validation in two longitudinal cohorts. *The Lancet*.

[151] Yang Y., Yi X., Cai Y., Zhang Y., Xu Z. (2022). Immune-associated gene signatures and subtypes to predict the progression of atherosclerotic plaques based on machine learning. *Frontiers in Pharmacology*.

[152] Sharma D., Gotlieb N., Farkouh M. E., Patel K., Xu W., Bhat M. (2022). Machine learning approach to classify cardiovascular disease in patients with nonalcoholic fatty liver disease in the UK Biobank Cohort. *Journal of the American Heart Association*.

[153] Chen Z., Yang M., Wen Y., Jiang S., Liu W., Huang H. (2022). Prediction of atherosclerosis using machine learning based on operations research. *Mathematical Biosciences and Engineering*.

[154] Jones G., Parr J., Nithiarasu P., Pant S. (2021). Machine learning for detection of stenoses and aneurysms: application in a physiologically realistic virtual patient database. *Biomechanics and Modeling in Mechanobiology*.

[155] Jiang Y., Yang Z.-G., Wang J. (2022). Unsupervised machine learning based on clinical factors for the detection of coronary artery atherosclerosis in type 2 diabetes mellitus. *Cardiovascular Diabetology*.

[156] Ross E. G., Shah N. H., Dalman R. L., Nead K. T., Cooke J. P., Leeper N. J. (2016). The use of machine learning for the identification of peripheral artery disease and future mortality risk. *Journal of Vascular Surgery*.

[157] Fan J., Chen M., Luo J. (2021). The prediction of asymptomatic carotid atherosclerosis with electronic health records: a comparative study of six machine learning models. *BMC Medical Informatics and Decision Making*.

[158] Cox M., Reid N., Panagides J. C. (2022). Interpretable machine learning for the prediction of amputation risk following lower extremity infrainguinal endovascular interventions for peripheral arterial disease. *CardioVascular and Interventional Radiology*.

[159] Gao J.-M., Ren Z.-H., Pan X. (2022). Identifying peripheral arterial disease in the elderly patients using machine-learning algorithms. *Aging Clinical and Experimental Research*.

[160] Kumar P. R., Priya M. (2014). Classification of atherosclerotic and non-atherosclerotic individuals using multiclass support vector machine. *Technology and Health Care*.

[161] Park S., Ahn J. W., Jo Y. J. (2020). Label-free tomographic imaging of lipid droplets in foam cells for machine-learning-assisted therapeutic evaluation of targeted nanodrugs. *ACS Nano*.

[162] Dai L., Zhou Q., Zhou H. (2021). Deep learning-based classification of lower extremity arterial stenosis in computed tomography angiography. *European Journal of Radiology*.

[163] Afzal N., Sohn S., Abram S., Liu H., Kullo I. J., Arruda-Olson A. M. Identifying peripheral arterial disease cases using natural language processing of clinical notes.

[164] Flores A. M., Demsas F., Leeper N. J., Ross E. G. (2021). Leveraging machine learning and artificial intelligence to improve peripheral artery disease detection, treatment, and outcomes. *Circulation Research*.

[165] Kampaktsis P. N., Emfietzoglou M., Al Shehhi A. (2023). Artificial intelligence in atherosclerotic disease: applications and trends. *Frontiers in Cardiovascular Medicine*.

[166] Johnson K. W., Torres Soto J., Glicksberg B. S. (2018). Artificial intelligence in cardiology. *Journal of the American College of Cardiology*.

[167] Karatzia L., Aung N., Aksentijevic D. (2022). Artificial intelligence in cardiology: hope for the future and power for the present. *Frontiers in Cardiovascular Medicine*.

[168] Van den Eynde J., Lachmann M., Laugwitz K. L., Manlhiot C., Kutty S. (2023). Successfully implemented artificial intelligence and machine learning applications in cardiology: state-of-the-art review. *Trends in Cardiovascular Medicine*.

[169] Visco V., Ferruzzi G. J., Nicastro F. (2021). Artificial intelligence as a business partner in cardiovascular precision medicine: an emerging approach for disease detection and treatment optimization. *Current Medicinal Chemistry*.

[170] Seetharam K., Balla S., Bianco C. (2022). Applications of machine learning in cardiology. *Cardiology and Therapy*.

[171] Coorey G., Figtree G. A., Fletcher D. F. (2022). The health digital twin to tackle cardiovascular disease—a review of an emerging interdisciplinary field. *NPJ Digital Medicine*.

[172] Corral-Acero J., Margara F., Marciniak M. (2020). The ’Digital Twin’ to enable the vision of precision cardiology. *European Heart Journal*.

[173] Visvikis D., Lambin P., Beuschau Mauridsen K. (2022). Application of artificial intelligence in nuclear medicine and molecular imaging: a review of current status and future perspectives for clinical translation. *European Journal of Nuclear Medicine and Molecular Imaging*.

[174] Krittanawong C., Johnson K. W., Choi E. (2022). Artificial intelligence and cardiovascular genetics. *Life*.

[175] Madan N., Lucas J., Akhter N. (2022). Artificial intelligence and imaging: opportunities in cardio-oncology. *American Heart Journal Plus: Cardiology Research and Practice*.

[176] Sadler D., Okwuosa T., Teske A. J. (2022). Cardio oncology: digital innovations, precision medicine and health equity. *Frontiers in Cardiovascular Medicine*.

[177] Martinez D. S.-L., Noseworthy P. A., Akbilgic O. (2022). Artificial intelligence opportunities in cardio-oncology: overview with spotlight on electrocardiography. *American Heart Journal Plus: Cardiology Research and Practice*.

[178] Vobugari N., Raja V., Sethi U., Gandhi K., Raja K., Surani S. R. (2022). Advancements in oncology with artificial intelligence—a review article. *Cancers*.

[179] Rezayi S., Kalhori S. R. N., Saeedi S. (2022). Effectiveness of artificial intelligence for personalized medicine in neoplasms: a systematic review. *BioMed Research International*.

[180] Nedios S., Iliodromitis K., Kowalewski C. (2022). Big data in electrophysiology. *Herzschrittmachertherapie + Elektrophysiologie*.

[181] Nedadur R., Wang B., Tsang W. (2022). Artificial intelligence for the echocardiographic assessment of valvular heart disease. *Heart*.

[182] Subramanian M., Wojtusciszyn A., Favre L. (2020). Precision medicine in the era of artificial intelligence: implications in chronic disease management. *Journal of Translational Medicine*.

[183] Harrison J. R., Mistry S., Muskett N., Escott-Price V., Brookes K. (2020). From polygenic scores to precision medicine in alzheimer’s disease: a systematic review. *Journal of Alzheimer’s Disease*.

